# Establishment of Quality Control Standard and Efficacy Evaluation of Zhiqingshu Lotion Compound Preparation

**DOI:** 10.1155/2022/2351366

**Published:** 2022-03-14

**Authors:** Benren Tan, Yichun Huang, Jinkun Zheng, Xiaomei Xu, Jian Xiao, Yanlin Liu

**Affiliations:** ^1^The Affiliated Yuebei People's Hospital of Shantou University Medical College, Shaoguan, Guangdong 512026, China; ^2^Shaoguan Institute for Food and Drug Control, Shaoguan, Guangdong 512028, China

## Abstract

**Objective:**

To establish the quality standard of Zhiqingshu lotion by high-performance liquid chromatography (HPLC).

**Methods:**

HPLC was used to determine emodin, chrysophanol, caffeic acid, and berberine hydrochloride content, key water-soluble components of rhubarb, dandelion, and Phellodendron amurense in Zhiqingshu lotion. The macrophage inflammation model was used to analyze the anti-inflammatory effects of Zhiqingshu lotion.

**Results:**

HPLC results showed that the contents of emodin, chrysophanol, caffeic acid, and berberine hydrochloride in Zhiqingshu lotion were 7.93 ± 2.25, 20.85 ± 4.27, 48.9 ± 6.79, and 58.4 ± 10.3 *μ*g/mL, respectively. Moreover, RT-qPCR results showed that different concentrations of Zhiqingshu lotion significantly reduced the expression of inflammatory factor tumor necrosis factor- (TNF-) *α* and interleukin- (IL-) 1*β* in lipopolysaccharide-induced macrophages.

**Conclusion:**

HPLC could quantitatively and qualitatively analyze and identify the main components of Zhiqingshu lotion as rhodopsin, rhodopsin, caffeic acid, and berberine hydrochloride. And Zhiqingshu lotion has an excellent anti-inflammatory effect. This method was simple and reliable and could be used for the identification of the ingredients and content of Zhiqingshu lotion, thus improving the quality control of the drug.

## 1. Introduction

Zhiqingshu lotion (ZQSL) is a traditional Chinese medicine compound formula developed based on the theory of traditional Chinese medicine. The preparation is concentrated and refined from various Chinese herbal medicines, including rhubarb, dandelion, Phellodendron amurense, and myrrh. In traditional Chinese medicine treatment, it has the effects of clearing away heat and detoxification, drying dampness and relieving itching, promoting qi and promoting blood circulation, and reducing swelling and pain [1]. It is mainly used to treat inflammatory external hemorrhoids, hemorrhoid incarceration, and other diseases [2–4]. The quality of traditional Chinese medicine compound prescriptions is essential in clinical treatment. Therefore, it is extremely important to strengthen the quality control and work implementation of traditional Chinese medicine preparations, improve the safety of the clinical medication, and ensure the reliability of the efficacy [5]. At present, the reference source for the quality standard specification for ZQSL is the Guangdong Province Preparation Registration Standard of Medical Institutions (Guangdong ZB20111771). However, this standard does not establish a content determination standard, only involving the pharmaceutical properties of the drug and the thin-layer chromatography identification of the main drug rhubarb [1, 6]. There are still big restrictions on the quality control and pharmaceutical efficacy evaluation of ZQSL.

Because of its high resolution, fast analysis speed, wide application range, no damage to the analyzed components, different detectors that can be configured according to the structural characteristics of the required detected compounds, etc., high-performance liquid chromatography (HPLC) technology has become the most widely used method in the quality control and fingerprint study of Chinese herbal medicine [7]. To improve the quality of ZQSL and enhance its efficacy and safety in clinical application, this study intends to refer to the Chinese Pharmacopoeia 2020 edition I criteria and related literature and use HPLC to qualitatively and quantitatively detect ZQSL key water-soluble components emodin, chrysophanol, caffeic acid, and berberine hydrochloride of rhubarb, dandelion, and Phellodendron amurense, to establish the quality standard of ZQSL and evaluate the efficiency of ZQSL with the macrophage inflammation model. The curative effect of the drug provides a reference for improving the quality and efficacy of ZQSL.

## 2. Experimental Materials

### 2.1. Instruments

High performance liquid chromatography (Aglient 1260), Shimadzu SHIMADZU (LC-30AD). Chromatographic column: Kromasil 100-5-C18 (5 *μ*m,250 mm × 4.6 mm), Agilent ZORBAX RX-C18 (5 *μ*m,250 mm × 4.6 mm). Electronic balance (METTLE TOLEDO AG135, precision 0.00001 g). HT-300BQ ultrasonic cleaner (Jining Hengtong), GoodLook-2000 high picture quality automatic thin-layer chromatography imaging system (Shanghai Kezhe Biochemical Technology Co., Ltd.).

### 2.2. Reagents and Standards

Emodin standard (batch number: 110756-200110, purity: 99.6%), chrysophanol standard (batch number: 110796-201319, purity: 96.8%), caffeic acid standard (batch number: 110885-201703, purity: 99.7%), and berberine hydrochloride standard (batch number: 110713-201814, purity: 86.7%) were purchased from the National Institute for Food and Drug Control. ZQSL (preparation from Yuebei People's Hospital, batch number: 20200617). Acetonitrile and methanol were chromatographically pure (TEDIA Company). Trichloromethane, ethyl acetate, and formic acid were purchased from Guangzhou Chemical Analysis Factory, all analytically pure. Water was redistilled water. Fetal bovine serum, 1% penicillin-streptomycin, and DMEM medium were purchased from Gibco, USA.

### 2.3. Preparation of HPLC Samples

Appropriate amounts of emodin, chrysophanol standard, caffeic acid standard, and berberine hydrochloride standard were accurately weighed and added with 50% methanol to prepare reference solution at concentrations of 0.7105, 0.2032, and 0.1852 mg·mL^−1^, respectively. About 20 mL of ZQSL was precisely measured, placed in a 50 mL measuring flask with methanol added to dilute to the mark. The mixture was shaken well and filtered, and the filtrate was taken to obtain the test solution. According to the prescription ratio of ZQSL, the negative medicines lacking dandelion, Phellodendron amurense, and rhubarb were prepared as the research objects, and the negative control solution required for the experiment was prepared according to the preparation method of the prescription drug solution provided.

### 2.4. HPLC Conditions

The octadecylsilane-bonded silica gel was used as the filler. After repeated pretests, the gradient elution was determined, with acetonitrile as the mobile phase A and 1% phosphoric acid as the mobile phase B. The elution gradient is shown in Table 1.

### 2.5. Quantitative Method Validation

0.1, 0.2, 0.5, 1, and 2 mL of emodin, chrysophanol, caffeic acid, and berberine hydrochloride reference solutions were, respectively, pipetted into five 10 mL volumetric flasks. Methanol was used to dissolve and dilute to the labeled scale and gently shaken well to obtain the required diluted methanol solution. 10 *μ*L of each solution was precisely pipetted and performed linear regression analysis with the content of the reference substance as horizontal axis (*X*) and the peak area as vertical axis (*Y*) according to the chromatographic conditions. An appropriate amount of the negative control solution was precisely pipetted, the sample determination was carried out according to the chromatographic conditions, and the anti-interference test was carried out. 10 *μ*L of the reference solution was precisely pipetted, respectively; according to the prepared chromatographic conditions, samples were consecutively injected 5 times to determine the content and conduct precision testing. 6 bottles of ZQSL were taken to prepare the test solution, injected the sample for determination, and verified the repeatability.

### 2.6. Cell Culture and Processing

Mouse peritoneal macrophages (RAW264.7) were purchased from ATCC in the United States and cultured in DMEM medium containing 10% fetal bovine serum and 1% penicillin-streptomycin and placed for incubation in a 37°C and 5% CO_2_ incubator. ZQSL was accurately measured to prepare solutions with 0, 10, 20, and 40 mg/mL concentrations. After digesting and counting the RAW-264.7 cells in the logarithmic growth phase, they were seeded in a 6-well plate at a density of 1 × 10^5^ cells/well. After the cells adhered to the wall, they were pretreated with ZQSL for 2 h, and then, lipopolysaccharide (LPS) was added [8, 9]. The cells were collected 24 h later, and the levels of tumor necrosis factor- (TNF-) *α* and interleukin- (IL-) 1*β* in the cells were detected.

### 2.7. Quantitative Reverse Transcription-Polymerase Chain Reaction (RT-qPCR)

The total cellular RNA was extracted using the TRizol method. After NanoDrop detected the concentration and purity of the RNA, cDNA was prepared according to the primer reverse transcription kit (Thermo, USA). The mRNA expression levels of TNF-*α* and IL-1*β* were detected according to the instructions of the SYBR GREEN kit (TaKaRa, Japan). GAPDH was used as the internal reference control, and three replicates were set up in the experiment. The data from qRT-PCR were used to calculate the relative expression of the target gene using the 2 ^−*ΔΔ*Ct^ method. The primer sequences are shown in Table 2.

### 2.8. Statistical Analysis

Statistical analysis was performed using the SPSS 22.0 software. An independent sample *t*-test analyzed the comparison between groups, and the results were expressed as mean ± standard deviation (SD). *P* < 0.05 was used as the significant difference judgment criteria.

## 3. Results

### 3.1. HPLC Methodological Investigation

Furthermore, HPLC was used to quantitatively analyze the presence of emodin, chrysophanol, caffeic acid, and berberine hydrochloride in ZQSL. First, the methodological investigation of the HPLC method was carried out, and the results showed that emodin (*Y* = 39748*x* + 5398.4, *r* = 0.9999), chrysophanol (*Y* = 51553*x* + 13753, *r* = 0.9999), caffeic acid (*Y* = 2.8628 × 10^4^*x* + 5.6062 × 10^3^, *r* = 0.9983), and berberine hydrochloride (*Y* = 1.8153 × 10^4^*x* + 4.4639 × 10^3^, *r* = 1.000) showed a good linear relationship. The precision test results showed that the relative standard deviation (RSD) of emodin, chrysophanol, caffeic acid, and berberine hydrochloride was 0.13%, 0.31%, 0.42%, and 0.32% (*n* = 5), respectively, indicating that the instrument had good precision. The repeatability test showed that the RSD of emodin, chrysophanol, caffeic acid, and berberine hydrochloride was 0.56%, 0.26%, 0.79%, and 0.68%, respectively, indicating that the method had good repeatability (Table 3).

### 3.2. HPLC Method Can Quantify Emodin, Chrysophanol, Caffeic Acid, and Berberine Hydrochloride Contents in ZQSL

The anti-interference experiment results show no corresponding chromatographic peaks at the peak positions of emodin, chrysophanol, caffeic acid, and berberine hydrochloride in the negative solution. The peak time of emodin, chrysophanol, caffeic acid, and berberine hydrochloride in the control solution did not overlap, indicating an absence of interference in the peak position of the sample. HPLC was used to detect the key components of the main traditional Chinese medicines in ZQSL, and the results showed that the contents of emodin, chrysophanol, caffeic acid, and berberine hydrochloride were 7.93 ± 2.25, 20.85 ± 4.27, 48.9 ± 6.79, and 58.4 ± 10.3 *μ*g/mL (Figures 1 and 2).

### 3.3. ZQSL Has Good Anti-inflammatory Effects

The anti-inflammatory effect of ZQSL was further studied to evaluate the reliability of the quality standard method established in this study. The results (Figure 3) showed that after LPS treatment, the levels of TNF-*α* and IL-1*β* in RAE264.7 cells increased significantly. However, the release of inflammatory cytokines TNF-*α* and IL-1*β* in the cells was inhibited by adding ZQSL in a dose-dependent manner. The results show that ZQSL has good anti-inflammatory effects and further show that TLC combined with HPLC was feasible for ZQSL quality control.

## 4. Discussion

ZQSL has been widely used clinically due to its functions of clearing away heat, detoxifying, reducing swelling, and relieving pain [1]. However, the current quality standard definition of ZQSL is relatively shallow. The quality control effect is low with the nondefined composition content of the medicine, so there are big problems in its quality control. Our laboratory [1] tested emodin and chrysophanol content in ZQSL by HPLC in the early stage and achieved good results. However, emodin and chrysophanol are only the main ingredients in one of the contributing medicines and cannot comprehensively reflect the quality of ZQSL. Therefore, it is necessary to establish a complete and comprehensive treatment standard for ZQSL. Rhubarb, dandelion, and Phellodendron amurense are the three main components of ZQSL, which have essential functions such as clearing away heat and detoxification, diuresis, and drying dampness [10], and play an important role in the efficacy of the drug. However, HPLC is more widely used in traditional Chinese medicine quality control [11]. Therefore, this study adopted HPLC to qualitatively and quantitatively detect the content of key water-soluble components chlorogenic acid, caffeic acid, and berberine hydrochloride. It shows that the chromatographic method established in this study has strong anti-interference and easy operation and can be widely promoted and applied.

In terms of content determination, traditional Chinese medicine compound preparations are often multisystem and complex in components and often have water-soluble, fat-soluble, and other main components. In this study, by referring to the 2020 edition of the Chinese Pharmacopoeia and related literature, combined with the analysis of the prescription components of ZQSL, it was found that the main water-soluble ingredients were emodin, chrysophanol, caffeic acid, and berberine hydrochloride. After repeated experiments, using methanol, acetonitrile, and 1% phosphoric acid solution as mobile phases [12–15], gradient elution was used, the chromatographic peak shapes of the three water-soluble components were symmetrical, and the obtained separation effect was the best with no interference in the negative solution control. The experimental results show that the determination method was feasible. The results of this study showed that the contents of emodin, chrysophanol, caffeic acid, and berberine hydrochloride in ZQSL were 7.93 ± 2.25, 20.85 ± 4.27, 48.9 ± 6.79, and 58.4 ± 10.3 *μ*g/mL, respectively. Based on the previous experimental basis for determining the fat-soluble components emodin and chrysophanol in ZQSL, it is of positive significance to increase the determination of water-soluble components for the quality control and quality standard improvement of ZQSL.

In addition, studies have shown that ZQSL has an excellent therapeutic effect in the treatment of inflammatory hemorrhoids [2, 16], so we further verified its anti-inflammatory effect through in vitro cell models and provided therapeutic support for quality control methods and provided a basis for further study of its mechanism of action. Studies have shown that TNF-*α* is a proinflammatory cytokine that can increase the phagocytic ability of neutrophils and promote cell proliferation and differentiation [17–19]. Cytokine IL-1*β* mediates inflammatory response and can induce the expression of iNOS and other inflammatory factors [20–22]. This study shows that ZQSL has an anti-inflammatory effect by inhibiting the proinflammatory factors TNF-*α* and IL-1*β*, reducing inflammation through direct or indirect effects. However, the anti-inflammatory effect of ZQSL needs to be further confirmed through clinical trials and more in vitro cellular experiments.

## 5. Conclusion

In this study, the quality control of ZQSL was carried out. The qualitative identification methods of rhubarb, dandelion, and Phellodendron amurense in the preparation were established as well as the quantitative analysis methods of emodin, chrysophanol, caffeic acid, and berberine hydrochloride. The efficacy of ZQSL under this quality standard was verified through in vitro anti-inflammatory experiments. The above methods are highly specific, accurate, and reliable and provide a reference for formulating the quality standard of ZQSL.

## Figures and Tables

**Figure 1:** Determination of emodin and chrysophanol content in Zhiqingshu lotion: (a) HPLC chromatogram of emodin and chrysophanol reference substance; (b) HPLC chromatogram of Zhiqingshu lotion test solution; (c) HPLC chromatogram of the negative reference substance.

**Figure 2:** Determination of caffeic acid and berberine hydrochloride content in Zhiqingshu lotion: (a) HPLC chromatogram of caffeic acid and berberine hydrochloride reference substance; (b) HPLC chromatogram of Zhiqingshu lotion test solution; (c) HPLC chromatogram of the negative reference substance.

**Figure 3:** The effect of Zhiqingshu lotion on TNF-*α* and IL-1*β* levels in RAW264.7 cells treated with LPS. ^∗∗^*P* < 0.01 vs. the first group, #*P* < 0.05 vs. the second group.

**Table 1:** Mobile phase elution gradient.

Time (min)	8	15	30	50	60	70
Acetonitrile	10	18	25	30	40	80
1% phosphate buffer solution	90	82	75	70	60	20

Column temperature: 30°C. Flow rate: 1 mL·min^−1^. Detection wavelength: 324 nm. Injection volume: 10 *μ*L. The number of theoretical plates calculated as chlorogenic acid should not be less than 3000.

**Table 2:** Primer sequences.

Primer	Sequence (5′-3′)
TNF-*α*	F: CTTCTGCCTGCTGCACTTTG
	R: GTCACTCGGGGTTCGAGAAG
IL-1*β*	F: GTACCTGTCCTGCGTGTTGA
	R: GGGAACTGGGCAGACTCAAA
GAPDH	F: CATCACTGCCACCCAGAAGACTG
	R: ATGCCAGTGAGCTTCCCGTTCAG

**Table 3:** HPLC methodological investigation.

	Linear regression	Precision	Repeatability
Emodin	*Y* = 39748*x* + 5398	0.13%	0.56%
Chrysophanol	*Y* = 51553*x* + 13753	0.31%	0.26%
Caffeic acid	*Y* = 2.8628 × 10^4^*x* + 5.6062 × 10^3^	0.42%	0.79%
Berberine hydrochloride	*Y* = 1.8153 × 10^4^*x* + 4.4639 × 10^3^	0.32%	0.68%

## Data Availability

The data used to support the findings of this study are available from the corresponding author upon request.
